# Social Media Big Data Analysis: Towards Enhancing Competitiveness of Firms in a Post-Pandemic World

**DOI:** 10.1155/2022/6967158

**Published:** 2022-03-03

**Authors:** Abdelaziz Darwiesh, Mohammed. I Alghamdi, A. H. El-Baz, Mohamed Elhoseny

**Affiliations:** ^1^Department of Mathematics, Faculty of Science, Damietta University, New Damietta, Egypt; ^2^Department of Engineering and Computer Sciences, Al-Baha University, Al Baha, Saudi Arabia; ^3^Department of Computer Science, Faculty of Computers and Artificial Intelligence, Damietta University, New Damietta, Egypt; ^4^University of Sharjah, Sharjah, UAE

## Abstract

In this paper, we proposed an advanced business intelligence framework for firms in a post-pandemic phase to increase their performance and productivity. The proposed framework utilizes some of the most significant tools in this era, such as social media and big data analysis for business intelligence systems. In addition, we survey the most outstanding related papers to this study. Open challenges based on this framework are described as well, and a proposed methodology to minimize these challenges is given. Finally, the conclusion and further research points that are worth studying are discussed.

## 1. Introduction

COVID-19 is one of the most consequential pandemics that have a big impact on societies, firms, and the global economy since the 1930's great depression [1]. During the pandemic, many firms have been forced to close or minimize their operations and those who continue deployed new digital systems for communications to adapt to the COVID-19 environment. Studies prove that digital technologies such as social media, information systems technology, and cloud-based infrastructure played an important role in response to the pandemic, and they are no longer used by firms but by societies [2]. In a post-pandemic, the competitiveness between firms will increase due to the periods of lockdowns during the pandemic and the future is for who can be equipped with up-to-date methodologies and technologies [3].

Business intelligence systems have been pivotal in the developing process and increasing competitiveness since they appeared in 1865 [4]. In the post-pandemic and with the widespread of new technologies like social media and big data, these systems became inefficient. At present, billions of people around the world use social media platforms daily to share their interests, opinions, activities, etc. [5]. Consequently, a huge amount of data is produced more than ever before and has different characteristics such as big volume, big velocity, big variety, and big value [6]. So, it is impossible to benefit from these big data by using classical business intelligence systems, and the evolution to modern systems based on new technologies became an urgent necessity for firms, specifically in a post-pandemic phase [7].

Social media big data analysis is a promised solution to develop classical business intelligence systems and make better decisions for firms and organizations. Depending on the Scopus database, we find that the number of publications in social media big data analysis is very low. In the period from 2012 to 2016, the number of publications ranged from 1 to 99 publications. This number increased more and reached up to 200 publications in the period from 2017 to 2021 as shown in Figure 1.

In these publications, the number of articles is greater than that of conference papers and book chapters, and the maximum number of articles reached 123 in 2020, which is shown in detail in Figure 2.

Also, the number of funded projects in this area is very low although it is increasing year by year as shown in Figure 3.

This paper provides an up-to-date business intelligence framework based on social media big data analysis to increase the capabilities of firms in competitiveness in the post-pandemic phase and makes their performance more trendy and powerful. Besides, this paper surveys the most important papers mentioned in Q1 or Q2 journals that related to our study. Moreover, we present the common challenges of the new framework and propose a new methodology to decrease these challenges. In the last, some research points are proposed for further research.

The rest of the paper is as follows: in Section 2, a survey and summary for research articles that related to our study is included; the new framework is presented in Section 3; in Sections 4 and 5, the basic challenges of the new framework and the proposed methodology to overcome these challenges are addressed; and finally, the conclusion is summarized, and new research points are provided in Section 6.

## 2. Literature Review

Social media, big data analysis, and business intelligence have been hot research topics in recent years. Big data analysis has a great impact on the development of firms, and many researchers utilize it in intelligent information systems to develop the decision-making process [8, 9]. Also, social media in business intelligence has attracted broad interest because of the enormous effect on the competitiveness of business [10]. The explosion in data generation in social media platforms directed the attention from traditional tools in data management and warehousing into big data technologies [11]. This literature is divided into three parts: big data analysis for business intelligence, social media for business intelligence, and social media with big data analysis. A summary of the literature review is given in Table 1.

### 2.1. Big Data Analysis for Business Intelligence

Big data has appeared in business intelligence since 2011 [12]. Big data as a technology and platform played a vital role in enhancing the productivity and capabilities of the firms [13]. It can help business intelligence activates in creating, delivering, and capturing customer value, which would lead to better making decisions for customers and firms [14]. Many papers discussed the leveraging big data analysis for business intelligence [4, 15–23].

In [4], the authors stated that big data impacts business intelligence through data analysis and new trends such as fast analysis and data science are emerged in business intelligence. In [15], a special issue presented the evolution and the applications of business intelligence and big data. In [19], a special issue introduced the research areas related to big data and business intelligence and addressed the challenges that need to be solved. In [22], the authors constructed a predictive churn model by using big data analytics tool to study the client retirement journey path. In [20], the authors found an expansion in the utilization of big data analysis as a tool in hospitality and tourism management.

### 2.2. Social Media for Business Intelligence

*Social Media, an Evolution of Communications in the 21st Century*. It has changed the lifestyle of people and made the world as a small city. People can communicate easily from any place and share their opinions and experiences with others [24]. Firms and organizations are adopting social media to acquire information from the users of social media websites to gain valuable insights for improving the quality of products, building brands, and increasing sales [25, 26]. Many authors discussed the deployment of social media in business intelligence [27–33].

In [27], the authors provided a systematic review of the research papers related to this domain. In [29], the authors found a positive relationship between social media analytic practices, customer engagement, and business performance. In [28], the authors proposed social business intelligence as a new research area for academia and industry. In [30], the authors built a prediction model to measure brand personality from social media users such as consumers, employees, and organizations. In [23], the authors studied the multivariate Gaussian distribution with the power-law distribution to detect the user's abnormal emotions of users in microblogs.

### 2.3. Social Media with Big Data Analysis

Due to the huge amount of users on social media platforms, massive and unstructured data are generating in relatively short timescales. It is necessary to analyze these data and obtain new insights. Different analysis as sentiment analysis and network analysis and several techniques as data mining and machine learning techniques can be involved to handle the growth of data generation in social media platforms [34]. Many papers study the integration between social media and big data analysis [35–41].

In [38], the authors presented a broad prescriptive of the big social media analytics research topic. They discussed the applications, state-of-the-art techniques, methods, and open research challenges related to this topic. In [35], the authors provided a systematic literature review of big data analysis in social network services between 2013 and 2020.

## 3. The Proposed Business Intelligence Framework for Firms

In this section, the proposed framework is shown in Figure 4. It describes several iterative steps that are beginning of formulation of the research problem statement, then entry and processing the data, then obtaining important insights that can be visualized and will be helpful in increasing the competitiveness of the firms in a post-pandemic, and developing smart applications, technologies, and approaches. The evaluation of the applied results is the last step, and then it leads to state a new research problem.

Firstly, the research problem that is under consideration is formulated. This helps in the following steps to choose the type of data that will be collected and the kind of analysis that will be performed on the data. The next step is the data entry that includes the determination of the potential social media platform such as Facebook, Twitter, and Instagram, and the type of selection data to collect it by using gathering data tools and making it available for further steps. The data have many types such as text, image, video, or sound and may be structured, semistructured, or unstructured. There are many tools to collect data from social media platforms as questionnaires, direct databases access to the company's servers, sanctioned API (application programming interface), Web crawlers, and deployment of custom application based on social media platforms [42, 43]. The following step is the data processing that includes preparing, storage, and analysis for the entry data. After gathering the data, it needs to be prepared to store in the big data warehouse, and then the analysis will be done. In the preparation process, the data are extracted, cleaned, transformed, and loaded [44]. The output of this process is homogeneous structure data that can be ready to store in big data warehouses.

Big data warehouses are proposed to store and process big data and support data models for analysis at different levels of detail. They differ from traditional data warehouses that support online analytical processing and are used by organizations to collect daily data to help them in the decision-making process [45]. Hive is considered as a big data warehouse that can facilitate querying and managing a huge amount of data that are stored in distributed storage systems. It is suited in a static data case that means no rapidly changing or no fast responses are needed. Also, NoSQL databases can be considered as a big data warehouse after transforming traditional data models into data models for NoSQL databases [46].

After storing data, the analysis process is ready to perform. In this process, big data frameworks such as Spark, Apache Hadoop, and smart tools to analyze social media content are conducted [47]. The analysis process includes deploying algorithms and methods to extract insights from the data entry. Machine learning and natural language processing (NLP) are the most commonly used techniques to make better analysis especially for textual data [48]. Various types of analysis can be performed such as descriptive analysis, predictive analysis, diagnostic analysis and prescriptive analysis, simulation, and optimization [49]. Besides, sentiment analysis, trend analysis, network analysis, and different analyses based on application such as market analysis, financial analysis, and crime analysis can be included.

In reaching this step, the extracted insights are visualized to help the decision-makers in firms and organizations in the decision-making process. The visualization step is necessary to convert the measured data to visualized data. Also, it is used as a presentation tool for illustration and explanation of results and has different forms such as charts and bars. Visual analytic techniques provide a quick and dynamic understanding of a tremendous amount of information in real time [46]. The findings of all previous steps lead to business development. This development includes enhancing the competitiveness between firms in a post-pandemic and smart technologies, applications, and approaches. Finally, the evaluation process for all findings is required. It helps us in assessing the decisions undertaken and discovering new problems.

## 4. Challenges and Current Issues for the Proposed Business Intelligence Framework

Today, social media platforms can be easily accessible through all over the world in real time. More than a billion users on different social media platforms create a huge amount of data through their daily activates such as posts, likes, and comments. This massive amount of data provides many opportunities and challenges for researchers and practitioners. It has different structures (unstructured, semistructured, structured) and many types (such as text, photo, video, and audio) that brought some challenges that need to be solved to obtain valuable insights [50]. In Figure 5, some of the most existing challenges are described. The challenges are divided into three parts: data entry challenges, data processing challenges, and data visualization challenges.

### 4.1. Challenges in Data Entry

Data entry has several challenges:

- Gathering data tools: building effective gathering data tools is a big challenge due to the different structures, types, and the huge amount and the velocity of creation data on social media platforms. In general, some of the challenges for the current gathering data tools are API handling, flexibility in scaling process, real-time report generation, generalization, and reliability [51]. Making appropriate data collection tool for each social media platform may be a good solution to solve this problem. For example, API is a good solution for Twitter, but in Facebook the privacy of users' data, long text of messages, and streaming data are still challenges for effective data collection tools.
- Data quality: as data are unstructured and collected from a wide range of users, the quality of data will be decreased. Data quality faces many challenges such as the difficulty of data integration due to the diversity of data sources that bring abundant data types and complex data structures, judging data quality within a reasonable amount of time due to huge amount of data, and timeliness of data is very short due to the fast change in data that require high technologies in processing and data quality standards [52]. Data cleaning and filtering techniques can deal with this issue [39, 53].
- Privacy: protecting the privacy of users on social media platforms is an important issue. Collecting the personal data of users by firms without striking a balance between the use of personal data and privacy concerns makes an untrusted environment. The balance is regarding to type of service, personal data, customers served, and regulatory environments. Some challenges are still open for privacy problems such as social identification and evaluation of test privacy-preserving services with real data [36]. Some solutions are given for this problem such as “k-anonymity” and “differential privacy” [36], but more efforts are still required.
- Validity: social media data may face some issues such as misinformation, fake accounts, and fake news. These issues make a bad effect on any analytical process, and the output insights will be biased; for example, the mislead public opinion that occurred during the 2016 US presidential election [54].  Section 5.3 works on solving validity issue. Besides, an ensemble machine learning approach through effective feature extraction is a considerable technique to classify fake news. It extracts the important features of fake news and then classified them using ensemble models with a high accuracy rate [55].

### 4.2. Challenges in Data Processing

Challenges in the stage of data processing are related to some characteristics of big data. Preparing, data warehousing, and analysis steps face the following challenges:

- Volume: social media platforms produce daily an enormous amount of data (e.g., Facebook generates daily more than 500 terabytes, over 2.5 petabytes per hour from Walmart customer transactions). Retrieval and processing this large scale of data is a challenge in itself and brought new challenges in data mining techniques [56]. Sections 5.2, 5.4, and 5.5 work on minimizing the volume of data that may be a good solution for this issue. In addition, analysis of dimensionality reduction techniques on big data such as linear discriminant analysis (LDA) and principal component analysis (PCA) is useful to reduce the complexity of high-dimensional data sets [57].
- Velocity: the generated data from social media platforms are of high speed and increase over time, which creates a big challenge. Real-time analysis is used to analyze data due to the velocity of data instead of batch analysis that is used early with low speed of data generation. The connected devices that share data are growing and accelerating the velocity [58].
- Variety: dealing with different types of data such as structured, semistructured, and unstructured in addition to several formats such as texts, images, videos, and audios is a major challenge. The captured data have enormous volume, are dissimilar, and do not follow a specific format (e.g., emails, tweets, images/videos/audios posted on social media sites). This diversity and heterogeneity decrease the quality of data and make managing and comprehending such data is a big challenge [56]. A proposed solution for this issue is mentioned in Section 5.2.
- Value: extracting value from all terabytes and petabytes of available data by using effective cost and reliable methods is a real challenge. It can transform firms and organizations to have more competitiveness in the global platform [59].
- Latency: it is one of the important factors for measuring system performance. Low latency refers to the quick system response to actions, which is a challenge in the case of large-scale data. It is considered a requirement for real-time analytics and modern businesses. It depends on storing and organizing large-scale data, processing the streaming data straight away, and performing effectively tasks with different priorities by using high capabilities of hardware and software [60]. Also, reducing the complexity of the data can lead to low latency. Other solutions can be included such as load balancing technique as in [61].
- Locality: in big data systems, the data are stored distributed in several physical locations. Most machine learning algorithms consider the data sets are located in the memory, and it is not applicable that make an issue in the data retrieval process [38].
- Availability: machine learning algorithms depend on the availability of the data set to make different tasks such as classifications, clustering, and prediction. In streaming data analysis, the data are not available and are arriving continuously [38].

### 4.3. Challenges in Data Visualization

Logically, the visual representation is more acceptable to a human rather than textual representative. For firms and organizations, the visualization process promotes capabilities, collaborations, and competitiveness. Visualization tools can display the obtained insights from various business perspectives. In the era of big data, visualization is important in identifying hidden patterns and trends in a vast amount of data and transforming it from useless data to useful and understandable. There are some challenges for big data visualization, which are as follows:

- Big data nature: due to the characteristics of big data mentioned in Section 4.2, the visualization process is a big challenge. Massive data, diversity, heterogeneity, high complexity, high dimensionality, and so on, make it difficult to conduct data visualization. Most of the current data visualization tools are poor in scalability, functionality, and response time. So, it is necessary to build effective real-time interactive visualization tools to make this process more flexible [62].
- Loss information: reduction approach that is used to decrease the dimensionality of data to make data visualization leads to loss information. This may affect badly the accurate and required data [63]. This problem can be solved when the complexity of big data is decreased, as in Section 5.5.
- High-performance requirements: graphical representation has two kinds, static and dynamic. In static visualization, lower visualization speed requirements need high-performance requirements [63].
- High rate of image change: this challenge is more significant in monitoring tasks when the user cannot react to the number of data changes or in its intensity on display. The simple decrease in changing rate cannot provide the target result because of the human reaction speed depending on it [63].
- Large image perception: data visualization methods are limited by the aspect ratio and resolution of the device and physical perception. Shown at once the growth of data volumes makes humans meet issues in understanding data and its analysis [63].
- Scalability and multilevel hierarchy: multilevel hierarchy approach is the main approach to many visual scalability problems. Scroll around deep multilevel hierarchy and finding an optimal resolution are real challenges for scalability analysis [64].

## 5. Suggested Methodology for Minimizing the Challenges of the Proposed Business Intelligence Framework

When you deal with the framework in Figure 4 and to minimize the previous challenges, we suggest a new approach that is shown in Figure 6. This approach focuses on solving the problems of the validity of data as in Step 5.3 and the complexity of big data as in Steps 5.2 and 5.5.

### 5.1. Data Collection

This step can be described by Algorithm 1.

### 5.2. Data Classification

This step is important to minimize the complexity of collected data such that big data may include different types of data. So, we consider the case of existence of three types of data (structured, unstructured, and semistructured) in Algorithm 2.

### 5.3. Data Scanning

This step is considered an important solution for validity problem by using the following procedure:

(1) Define criteria for the input data to determine the types of data that can be used in the required analysis. These types of data can be classified as follows:
  - Rejected data: it contains misinformation, fake account, and fake news
  - Acceptable data: it contains misinformation that can be imputed
  - Good data: it has good quality but is biased (not represent the population)
  - Very good data: it has good quality and is not biased but does not represent the actual opinions (due to freedom restrictions)
  - Perfect data: it does not have any of the mentioned previous problems
(2) Weight each input data due to its type, as shown in Table 2.
(3) Compare the weight of each input data with the defined criteria, when it is equal or greater to the defined criteria, then assign it to a big data warehouse, else delete the input data.

This procedure is very helpful because some analytics need to deal with a specific type of data such as campaign management and market management. Also, the selected data that have been assigned in the big data warehouse may have different types of data (e.g., perfect data and very good data with good data). So, the following inequality should be satisfied:

(1) $$\begin{array}{c} P_{\mathrm{Pr}}>P_{Vg}>P_{G}, \end{array}$$

where *P*_Pr_, *P*_*Vg*_, *P*_*G*_ are the portions of perfect, very good, and good data, respectively. The algorithm of this process can be described in Algorithm 3.

In addition to the above solution, other techniques can be involved such as an ensemble machine learning approach to deal with fake news. It extracts the important features of fake news and then classify them using an ensemble model with a high accuracy rate [55].

### 5.4. Feature Extraction

This step can be described by Algorithm 4.

### 5.5. Feature Selection

This step is a vital step with Step 5.2 in decreasing dimensionality of big data and that can be described by Algorithm 5.

Also, other solutions can be addressed here to decrease the complexity of big data such as analysis of dimensionality reduction techniques on big data. For example, linear discriminant analysis (LDA) and principal component analysis (PCA) are useful to reduce the complexity of high-dimensional data sets [57].

### 5.6. Data Mining

In this step, a suitable technique to obtain insights from the selected features is chosen.  Algorithm 6 describes how this step is working.

### 5.7. Visualization

This is the last step. Based on the previous steps, the challenges of the visualization process may be decreased more than before. Many techniques of visualization can be applied to the insights *Y* to make the best decisions *Z*.

## 6. Conclusion and Future Work

In a post-pandemic, firms have many challenges, and hence new methodologies and approaches need to be developed. We presented an advanced business intelligence framework to increase the competitiveness of the firms and make their performance trendy and powerful. This framework merges social media and big data analysis for business intelligence systems. Also, the most important research papers related to this study and published in Q1 and Q2 journals are surveyed. Moreover, we stated the challenges of the proposed approach and suggested a new methodology to reduce these challenges. Finally, many potential research points for further research are provided.

Many research points can be developed depending on the new framework. Business intelligence models, approaches, technologies, and applications will be impacted deeply through emerging social media and big data analysis for business intelligence systems specifically in a post-pandemic phase. Researchers can work on the mentioned challenges in Section 4 and propose new solutions for these challenges. Besides, many research points that can be studied as a further study include the following:

- Deploying social big data analysis intensely in finance. For example, risks in cryptocurrencies, stocks, and e-commerce can be identified, evaluated, and optimized by using social media big data analysis.
- Crisis and risks prediction for many applications such as industry, political, culture, health care, and policy can be done by using social media big data analysis.
- Applying social media big data analysis in computational social science to gain deep insights about the individual's behavior on social media platforms.
- Mapping social big data analysis for cartography and geographic information science that will be useful in many applications such as confronting terrorists and identifying their locations.
- Using social big data analysis in enabling B2B domain to maximize the profit of companies.
- Converting actions on social media platforms as like to buy action can be done by utilizing real-time data and big data analysis techniques.
- Finding a comprehensive solution to the hierarchy topic to enable aggregations of topics at different levels.
- Developing effective capturing, analysis, and visualizing tools to increase the benefits of business intelligence process.
- Identifying the characteristics of users on social media platforms by using big data analysis is helpful to increase the business profits.
- Analyzing how users rate the services qualitatively and quantitatively and give more interest to text reviews that has a potential effect on developing services and products.
- Studying social influence and information diffusion through different platforms simultaneously.

## Figures and Tables

**Figure 1:** Comparison between numbers of publications in the periods from 2012 to 2016 with the period from 2017 to 2021.

**Figure 2:** Types of publications, increasing from 2012 to 2021.

**Figure 3:** Funded projects, increasing from 2012 to 2021.

**Figure 4:** Advanced business intelligence framework for firms.

**Figure 5:** Challenges of the advanced business intelligence framework for firms.

**Figure 6:** A suggested solving challenges approach to the advanced business intelligence framework for firms.

**Algorithm 1:** Data collection algorithm.

**Algorithm 2:** Data classification algorithm.

**Algorithm 3:** Data scanning algorithm.

**Algorithm 4:** Feature extraction algorithm.

**Algorithm 5:** Feature selection algorithm.

**Algorithm 6:** Data mining algorithm.

**Table 1:** Summary of the literature review.


Author/s	Title	Year	Findings	Method	Application	Topic
Fuchs M, Höpken W, Lexhagen M	Big data analytics for knowledge generation in tourism destinations—A case from Sweden	2014	Creating the knowledge for determination of the tourism destination in Sweden by using big data analysis	Business intelligence approach	Tourism sector	Big data analysis for business intelligence
Babita G, Michael G, Barbara D	Business intelligence and big data in higher education: Status of a multi-year model curriculum development effort for business school undergraduates, MS graduates, and MBAs	2015	Developing models curricula for an elective business intelligence course at undergraduate and postgraduate programs	A multimethodological approach	Higher education sector	
Fan S, Lau R, Zhao J	Demystifying big data analytics for business intelligence through the lens of marketing mix	2015	Demystifying big data analytics for business intelligence	Lens of marketing mix framework	Marketing	
Sun Z, Sun L, Strang K	Big data analytics services for enhancing business intelligence	2018	The efficiency of using big data analytics in enhancing business intelligence and enterprise information systems	Big data analytics service-oriented architecture (BASOA) model	-	
Popovič A, Hackney R, Tassabehji R, Castelli M	The impact of big data analytics on firms' high value business performance	2018	The better utilization of big data analysis in decision-making process and the high value business performance	Interpretive qualitative approach	Manufacturing sector	
Rui H, Whinston A	Designing a social-broadcasting-based business intelligence system	2012	Framework of social-broadcasting-based BI systems that utilize real-time information	Sentiment analysis	Box office revenue	Social media for business intelligence
Lu Y, Wang F, Maciejewski R	Business intelligence from social media: A study from the VAST box office challenge	2014	The need for interactive tools to mine social media data	Visual analytics toolkit	Box office revenue	
Gallinucci E, Golfarelli M, Rizzi S	Advanced topic modeling for social business intelligence	2015	Expressive solution to model topic hierarchies	Meta-stars approach	—	
Sun X, Zhang C, Li G, Sun D, Ren F, Zomaya A, Ranjan R	Detecting users anomalous emotion using social media for business intelligence	2018	Modeling and analysis of the users' emotion of microblogs and detect abnormal emotion state	Multivariate Gauss distribution with the power-law distribution	—	
Yuheng H, Xu A, Hong Y, Gal D, Sinha V, Akkiraju R	Generating business intelligence through social media analytics: Measuring brand personality with consumer-, employee-, and Firm-generated content	2019	Prediction model to measure brand personality from multiple archival sources of social media content	A text analytics framework	Marketing	
Garg P, Gupta B, Dzever S, Sivarajah U, Kumar V	Examining the relationship between social media analytics practices and business performance in the Indian retail and IT industries: The mediation role of customer engagement	2020	Positive relationship between social media analytic practices, customer engagement, and business performance	Structural equation modeling analysis	Retail and IT sectors	
Immonen A, Pääkkönen P, Ovaska E	Evaluating the quality of social media data in big data architecture	2015	A new architectural solution to evaluate and manage the quality of social media data in each processing phase of the big data pipeline	Metadata management architecture	Marketing	Social media with big data analysis
Tsou MH	Research challenges and opportunities in mapping social media and big data	2015	Important research challenges and major opportunities for cartographers to process and visualize big data and social media	Short paper	Cartographic research	
Bello-Orgaza G, Jungb JJ, Camachoa D	Social big data: Recent achievements and new challenges	2015	A holistic view and insights for potentially helping to find the most relevant solutions that are currently available for managing knowledge in social media	Survey	—	
Felt M	Social media and the social sciences: How researchers employ big data analytics	2016	Outline some of the recent changes in social media data analysis, with a focus on twitter, specifically	Comparative case study	—	
Jimenez-Marquez JL, Gonzalez-Carrasco I, Lopez-Cuadrado JL, Ruiz-Mezcua B	Towards a big data framework for analyzing social media content	2019	A two-stage framework to tackle the problem of analysis text review and the additional features in raw data	Big data architectures	Tourism	

**Table 2:** Evaluation of types of data and the corresponding weight.

Type of data	Weight
Rejected data (*RD*)	−1
Acceptable data (*AD*)	0
Good data (*GD*)	1
Very good data (*VGD*)	2
Perfect data (*PD*)	3

## Data Availability

The analyzed data have been collected mainly from the Scopus database.
